This article has been retracted.

# Exploring the prophylactic role of soy isoflavones against polycystic ovarian syndrome

**DOI:** 10.1002/fsn3.2322

**Published:** 2021-07-09

**Authors:** Nishaf Manzar, Safwan Ahmad khan, Najum Fatima, Mehr un Nisa, Muhammad Haseeb Ahmad, Muhammad Inam Afzal, Hafiz Fahad Ullah Saeed, Muhammad Imran, Faqir Muhammad Anjum, Muhammad Sajid Arshad

**Affiliations:** ^1^ Department of Nutritional Sciences Government College University Faisalabad Pakistan; ^2^ Basic Health Unit (BHU) Faisalabad Pakistan; ^3^ District Head Quarter Hospital Chiniot Pakistan; ^4^ Department of Food Science Faculty of Life Sciences Government College University Faisalabad Pakistan; ^5^ Department of Biosciences COMSATS University Islamabad Islamabad Pakistan; ^6^ King Edward Medical University Lahore Pakistan; ^7^ Department of Diet and Nutritional Sciences University of Lahore Lahore Pakistan; ^8^ Vice Chancellor Secretariat University of the Gambia Banjul The Gambia

**Keywords:** digestibility, lipid profile, polycystic ovarian syndrome, soy isoflavones

## Abstract

Soy isoflavones (SI) have strong estrogenic effect in tissues by binding to estrogen receptors and might be beneficial for women with polycystic ovarian syndrome (PCOS) by reduction in testosterone, cholesterol, insulin, weight gain, inflammatory markers, and oxidative stress. The study was planned to examine the effect of various levels of SI on nutrient intake, digestibility, lipid profile, insulin, and reproductive hormones of estradiol valerate (4 mg/rat/IM) PCOS induced rat models. Thirty‐six Wistar 45 days old rats weighing 95 ± 5 g were divided into 4 groups, each having 9 rats: C (control: without SF), SF10 (SF 0.10 g/kg BW), SF15 (SF 0.15 g/kg BW), and SF20 (SF 0.20 g/kg BW). SF was given through the oral gavage. Food and water were offered ad libitum, and intake was recorded daily. During last week of trial, collected feces by total collection method and blood samples were used to calculate nutrient digestibility and biochemical analysis, respectively. Estrogen, progesterone, and prolactin were (*p* < .05) high in rats fed SF diet that was 4% and 30% increase from C, respectively. Insulin, testosterone, FSH, and LH were lowest in rats fed diet SF20. Significant (*p* < .05) reduction in cholesterol was observed in rats fed SF15 and SF20 as compared to C. Serum HDL was improved (*p* < .05) in all SIF_0.10_, SIF_0.15,_ and SIF_0.20_ in comparison with PC. Serum LDL was significantly reduced to 68.89 ± 4.36 (mg/dl) in SIF_0.20_ and to 108.20 ± 4.14 (mg/dl) in SIF_0.15,_ whereas insignificant reduction was observed in SIF_0.10_ as compared to PC. Highly significant reduction was noted in triglycerides level in SIF_0.20;_ however, significant reduction was observed in both SIF_0.10_ and SIF_0.15_ as compared to PC after 3 months of treatment with soy isoflavones.

## Abstract 2

The objective of this study was to investigate the effect of different levels of soy isoflavones on blood insulin, lipid, and reproductive hormones profile of the female rats with PCOS.

## 1 INTRODUCTION

In assessing the therapeutic effects of phytoestrogens, a clear dissimilarity must be made between foods having phytoestrogens and dietary supplements, as bioavailability, dosage, and physiological effect may vary critically (Setchell et al., 2001). The majority of phytoestrogens belong to a large group of substituted phenolic compounds known as flavonoids. Isoflavones are polyphenolic compounds that are almost exclusively produced by the members of the Fabaceae family. The major bioactive isoflavones are genistein and daidzein, which are derived mainly from soy and red clover (Ricci et al., 2010). In particular, soybeans are the richest sources of isoflavones in the human diet.

Isoflavones are identified to exhibit weak estrogen hormone‐like activity. Because isoflavones are not synthesized by the human endocrine system and can only be ingested or consumed in a diet or as a supplement, they are also called as “dietary estrogens” (Knight & Eden, 1996). In human body, estrogen is secreted primarily by the ovaries and in lesser quantities by the adrenal glands. The most active form of estrogen in the body is called estradiol. Estrogen puts its effects by binding to estrogen receptors within cells. These estrogen receptor complexes then combine with DNA to change the expression of estrogen‐responsive genes. For simulating the effects of estrogen in tissues, soy isoflavones as phytoestrogens can bind to estrogen receptors (Helmy et al., 2014).

As isoflavones and estradiol are contending for their binding on ERs, the effect of isoflavones also dependent on the level of endogenous estradiol. When there is high levels of endogenous estrogens, isoflavones may hinder full estrogen activity by conquering a part of the ERs. Alternatively, when there is low levels of endogenous estrogens, the estrogen activity of isoflavones may become evident (Lephart et al., 2003). As compared to 17‐β‐estradiol, the affinity of other isoflavones is 100–500 times lower. Isoflavones act against ERs, but their activity is lesser than that of 17‐β‐estradiol. At suitably high levels, the effect of isoflavones may approach the effect of endogenous 17‐β‐estradiol at its physiological level (Kuiper et al., 1997). For this reason, there is emerging trend of using isoflavones as an alternative or complement of HRT in postmenopausal women, particularly when long‐term administration is required (Davis et al., 1999). A number of studies indicate that soy, being high in isoflavones, can prevent illness and promote good health.

Soy isoflavones have number of benefits for women with PCOS such as reduction in testosterone, total cholesterol and LDL cholesterol, insulin, inflammatory markers, and oxidative stress (Khani et al., 2011). Polycystic ovary syndrome is the most common endocrine disorder among the women of reproductive age (Jalilian *et al.,* 2015).

In women with PCOS, insulin resistance is common and it causes lipoprotein disturbances that plays a role as predisposing factor for early development of diabetes, hyperlipidemia, and cardiovascular disease (Rizk et al., 2012). Two types of interventions, drug treatment and change in lifestyle with exercise and weight loss, are mostly used as therapeutic approaches for PCOS. The available common drugs are effective for PCOS, but they have side effects such as amenorrhea, overweight, decreased bone mineral density, and depression. Therefore, the use of nonpharmacological treatment methods is considered.

Using soy isoflavones as a nonpharmacological approach for PCOS patients, there is growing interest in how adding soy to the diet can help address metabolic syndrome and related health conditions are growing interest in how adding soy to the diet can help address metabolic syndrome and related health conditions. The effects of soy isoflavones have been studied by several researchers, and their biological activity related to estrogen receptor‐mediated mechanisms has been observed (Forouhari et al., 2013). Soy isoflavones being phytoestrogens are adaptogens. Under increased or decreased levels of estrogen, they can be beneficial. When isoflavones attached themselves to estrogen receptors, this hinders the effects of endogenous estrogen. Generally, phytoestrogens have about two percent of the strength of estrogens. Hence, when estrogen levels are high, switching a phytoestrogen for an estrogen means that there will be much less estrogenic activity at a given binding site. Conversely, if estrogen levels are low and estrogen‐binding sites are free, phytoestrogens that have almost two percent estrogen activity will bind with them and result in a total increase in total estrogenic effect (Barnes et al., 2000). Considering the above facts, the objective of this study was to investigate the effect of different levels of soy isoflavones on blood insulin, lipid, and reproductive hormones profile of the female rats with PCOS.

## 2 MATERIALS AND METHODS

This study was carried out in the Department of Food Science, Nutrition and Home Economics and Department of Pharmacy, Basic Sciences, Government College University, Faisalabad. The 36 Wistar albino female rats (45 days old), each with the weight 100 ± 10 g, which had 2 consecutive estrus cycles were bought from National Institute of Health, Islamabad. They were kept at 28 ± 1°C and 45%–55% relative humidity under 12‐hr light: 12‐hr dark cycle. According to Principles of Laboratory Animal Care (NIH), all animals were kept and treated. The approved experimental procedure by the Animal Ethical Committee was considered. Ad *libitum* diet and water were offered to the rats. *Isocaloric* and *isonitrogenous* diets were offered to the rats. The weekly intake of water and feed were monitored at least 1 week prior to treatments in order to regulate the amount of water drank per experimental animal. The soy isoflavones used for research were purchased from Xi'an Wharton Bio‐Tech, Co, Ltd, China.

### 2.1 Different levels of soy isoflavones

Thirty‐six PCOS induced Wistar female rats were used to observe the effect of different levels of isoflavones. The rats were divided into four groups (9 rats per group) named according to levels viz. PC (Positive control: without isoflavones), SIF_0.10_ (soy isoflavone: 0.10g/kg body weight), SIF_0.15_ (soy isoflavones: 0.15 g/kg body weight), and SIF_0.20_ (soy isoflavones: 0.20 g/kg body weight). These levels of soy isoflavones were given through oral gavage (Turner et al., 2012). All animals included in PC, SIF_0.10,_ SIF_0.15,_ and SIF_0.20_ were induced PCOS through single intramuscular injection of estradiol valerate (4 mg/rat/IM). In this in vivo experimental method, the rats were divided according to completely randomized design. In this study, total 39 rats were used and total 4 groups having 3 replicates.

The trial was of 3 months. The first 2 months were correction period followed by 1 month collection period. The 30 days before the experimental protocol, 36 rats were given a single intramuscular injection of 4 mg/rat estradiol valerate (Riedeldehaen, Germany) firstly mixed in 0.2 ml oil to induce PCOS (Ghasemzadeh et al., 2013). In the last week of study, all rats were bled to get blood samples to carry out biochemical and pathological analysis.

### 2.2 Feed and nutrient digestibility analysis

Digestibility of nutrients was measured by total collection method. All modified diets/feeds and feces were analyzed to calculate ash, moisture, crude protein, crude fat, crude fiber, nitrogen free extract, and dry matter content (AOAC, 2000).

Nutrient Digestibility (\% )=Nutrient intake‐Nutrient in feces×100

Feces sample was collected via designing the cages in such a way that collect samples accurately (Perline, 1971). Feces were stored at −20°C (Janczyk et al., 2007).

### 2.3 Biochemical analysis

In the end of trial, 5cc blood samples of all rats were drawn and prepared for biochemical analysis (Ghasemzadeh et al., 2013).

The plasma testosterone was estimated by method adopted by Yilmaz et al., (2005). Plasma estrogen levels were checked according to reference method of Stanczyk et al. (2007). The blood glucose was measured using ACCU Check Active^®^ Machine, and serum insulin was assessed by using Electrochemiluminescence immunoassay (Roche Diagnostics E170 insulin assay). The lipid profile was determined by the method described by cholesterol (Stockbridge et al., 1989), triglycerides (Annoni et al., 1982), high density lipoproteins (Assmann, 1979), and low density lipoproteins (McNamara et al., 1990).

### 2.4 Statistical analysis

The data obtained from all experimental sources were subjected to statistical analysis using completely randomized designed (CRD) according to the procedure described by Steel and Torrie (1997). Significant differences between the means of parameters were determined by using the Tukey test (*p* < .05).

## 3 RESULTS

### 3.1 Nutrient intake

The result showing the effects of different level of soy isoflavones on weight of PCOS induced rats is shown in Table 1. Slightly significant decrease was observed in dry matter intake when compared with PC. Values of crude protein intake were found to be decreased in all rats treated with soy isoflavones as 7.94 ± 0.21 in SIF_(0.10)_,8.31 ± 0.23 in SIF_(0.15),_ and 7.85 ± 0.24 in SIF_(0.20)_. Crude fiber intake was also significantly decreased in all groups with as low as 0.97 ± 0.16 in SIF _(0.15)_. Significant reduction in intake of ether extract and ash content of the feed was observed in all rats fed with different levels of soy isoflavones.

**TABLE 1:** Nutrient in take after administration of different levels of soy isoflavones in PCOS induced rats

Parameters	PC	SIF_(0.10)_	SIF_(0.15)_	SIF_(0.20)_
Dry matters intake (DMI) per day	26.61 ± 0.11^a^	24.71 ± 0.11^b^	24.65 ± 0.09^b^	24.41 ± 1.12^b^
Crude protein intake (%)	9.17 ± 0.24^a^	7.94 ± 0.21^b^	8.31 ± 0.23^b^	7.85 ± 0.24^c^
Crude fiber intake (%)	1.52 ± 0.16^a^	0.87 ± 0.16^bc^	0.97 ± 0.16^b^	0.87 ± 0.16^bc^
Ether extract intake EE	1.02 ± 0.59^a^	0.99 ± 0.71^b^	0.98 ± 0.71^b^	0.87 ± 0.68^c^
Ash (%)	3.95 ± 0.33^a^	2.53 ± 0.29^b^	2.36 ± 0.31^b^	2.34 ± 0.34^c^

Note

The values are means ± *SD* of three independent determinations. PC (positive control without isoflavones); SIF_0.10_ (soy isoflavones: 0.10 g/kg body weight); SIF_0.15_ (soy isoflavones: 0.15 g/kg body weight); SIF_0.20_ (soy isoflavones: 0.20 g/kg body weight).

### 3.2 Digestibility

The effects of different level of soy isoflavones on digestibility of PCOS induced rats were given in the Table 2. Dry matter digestibility was significantly decreased in all rats fed with various levels as 76.6 ± 0.64 in SIF_(o.15)_ and 70.2 ± 0.66 in SIF_(0.20)_. However, crude fiber digestibility was significantly decreased with 18% decreased SIF_(0.20)_. And significant reduction in values of ether extract was observed in all rats treated with different levels of soy isoflavones when compared with PC.

**TABLE 2:** Digestibility after administration of different levels of soy isoflavones in PCOS induced rats

Parameters	PC	SIF_(0.10)_	SIF_(0.15)_	SIF_(0.20)_
Dry matters digestibility (DMD)	75.89 ± 4.11^a^	69.12 ± 2.12^b^	71.21 ± 1.09^b^	63.19 ± 1.12^b^
Crude protein	82.7 ± 0.87^a^	76.6 ± 0.64^b^	77.1 ± 0.64^b^	70.02 ± 0.66^c^
Crude fiber	59.8 ± 0.68^a^	54.1 ± 0.71^b^	54.1 ± 0.71^b^	48.5 ± 0.74^c^
Ether extract	89.5 ± 0.78^a^	83.6 ± 0.51^b^	83.1 ± 0.48^b^	77.0 ± 0.98^c^

Note

The values are means ± *SD* of three independent determinations. PC (positive control without isoflavones); SIF_0.10_ (soy isoflavones: 0.10 g/kg body weight); SIF_0.15_ (soy isoflavones: 0.15 g/kg body weight); SIF_0.20_ (soy isoflavones: 0.20 g/kg body weight).

### 3.3 Weight changes

The result showing the effects of different level of soy isoflavones on weight PCOS induced rats is shown in the Table 3. Statistically significant reduction in final weight was observed in SIF_(0.20)_ as 72.5 ± 8.53 when compared with PC, after administration of soy isoflavones in PCOS induced female rats. In all rats treated with various levels of soy isoflavones, significant increase was observed in feed conversion ratio (FCR) with the maximum increase noted in SIF_(0.20)_ of about 20% as compared to PC.

**TABLE 3:** Weight/ht changes after administration of different levels of soy isoflavones in PCOS induced rats

Parameters	PC	SIF_(0.10)_	SIF_(0.15)_	SIF_(0.20)_
Initial weight	95.6 ± 1.52	97.2 ± 1.52	96.3 ± 1.52	97.7 ± 1.52
Weight after PCOS	124.6 ± 1.73	124.2 ± 1.73	127.2 ± 1.73	126.6 ± 1.73
Weight Gain First Month	30.0 ± 1.20	27.0 ± 1.20	30.0 ± 1.20	28.0 ± 1.20
Final Weight gain	93.4 ± 4.75^b^	79.4 ± 4.75^a^	77.2 ± 4.75^a^	72.5 ± 4.75^a^
Feed Conversion Ratio	15.4 ± 0.45^b^	17.7 ± 0.65^b^	18.2 ± 0.57^ab^	19.3 ± 0.69^a^

Note

The values are means ± *SD* of three independent determinations. PC (positive control without isoflavones); SIF_0.10_ (soy isoflavones: 0.10 g/kg body weight); SIF_0.15_ (soy isoflavones: 0.15 g/kg body weight); SIF_0.20_ (soy isoflavones: 0.20 g/kg body weight).

### 3.4 Reproductive hormones

The results showing the effects of different level of soy isoflavones on reproductive hormones of PCOS induced rats are shown in Table 4. In all rats treated with SIF_0.10_, SIF_0.15,_ and SIF_0.20,_ almost significant results were observed. Progesterone values were observed to be increased in all levels with maximum increase in SIF_0.20_ that is 13.21 ± 0.45 showing 30% increase from PC. Decrease in testosterone values was noted in all treatment levels. Notable change was seen in FSH/LH ratio, with increase in FSH values as noted maximum in SIF_0.10_ and SIF_0.20_, but is comparatively low in SIF_0.15,_ whereas remarkable decrease was observed in LH values with lowest most observed in SIF_0.20_ as (13.91 ± 0.67 mIU/ml). Increase was observed in prolactin values from PC in both SIF_0.10_ and SIF_0.20_ levels; however, reduction was noted in SIF_0.15_ (31.93 ± 1.04 ng/ml) from PC. In estrogen concentration, significant increase was observed in SIF_0.20,_ but no statistically significant change was noted in SIF_0.10_ and SIF_0.15_ from PC.

**TABLE 4:** Reproductive hormones after administration of different levels of soy isoflavones in PCOS induced rats

Parameters	PC	SIF_(0.10)_	SIF_(0.15)_	SIF_(0.20)_
Progesterone mg/mL	9.16 ± 0.45^b^	11.84 ± 0.48^a^	12.90 ± 0.43^a^	13.21 ± 0.45^a^
Testosterone ng/dL	112.70 ± 2.85^a^	97.34 ± 3.03^b^	89.29 ± 2.71^bc^	79.61 ± 2.85^c^
FSH mIU/mL	4.37 ± 0.32^a^	4.57 ± 0.34^a^	4.55 ± 0.30^a^	4.67 ± 0.32^b^
LH mIU/mL	18.18 ± 0.67^a^	16.50 ± 0.71^ab^	15.31 ± 0.64^bc^	13.91 ± 0.67^c^
Prolactin ng/mL	35.16 ± 1.10^bc^	37.55 ± 1.17^b^	31.93 ± 1.04^c^	44.29 ± 1.10^a^
Estrogen pg/mL	63.40 ± 2.88^b^	63.24 ± 3.05^b^	60.28 ± 2.73^b^	92.90 ± 2.88^a^

Note

The values are means ± *SD* of three independent determinations. PC (positive control without isoflavones); SIF_0.10_ (soy isoflavones: 0.10 g/kg body weight); SIF_0.15_ (soy isoflavones: 0.15 g/kg body weight); SIF_0.20_ (soy isoflavones: 0.20 g/kg body weight).

### 3.5 Lipid profile

Effects of different levels of soy isoflavones on lipid profile of PCOS induced rats are given in the Table 5. Significant reduction in cholesterol was observed in SIF_0.15_ and SIF_0.20_ as 141.60 ± 2.56 (mg/dl) and 127.56 ± 2.69 (mg/dl), while insignificant results were obtained in SIF_0.10_ 154.63 ± 2.86 (mg/dl) as compared to PC. Level of serum HDL was significantly improved in all SIF_0.10_, SIF_0.15,_ and SIF_0.20_ as 26.88 ± 1.59 (mg/dl), 32.40 ± 1.42 (mg/dl), and 53.44 ± 1.50 (mg/dl) in comparison with PC. Serum LDL was significantly reduced to 68.89 ± 4.36 (mg/dl) in SIF_0.20_ and 108.20 ± 4.14 (mg/dl) in SIF_0.15,_ whereas insignificant reduction was observed in SIF_0.10_ (127.75 ± 4.62 mg/dl) as compared to PC. Highly significant reduction was noted in triglycerides level in SIF_0.20_ as 115.00 ± 2.04 (mg/dl); however, significant reduction was observed in both SIF_0.10_ and SIF_0.15_ as compared to PC after 3 months of treatment with soy isoflavones.

**TABLE 5:** Lipid profile (mg/dl) and Insulin (mmol/L) after administration of different levels of soy isoflavones in PCOS induced rats

Parameters	PC	SIF_(0.10)_	SIF_(0.15)_	SIF_(0.20)_
Cholesterol	164.00 ± 2.69^a^	154.63 ± 2.86^a^	141.60 ± 2.56^b^	127.56 ± 2.69^c^
HDL	19.89 ± 1.50^c^	26.88 ± 1.59^b^	32.40 ± 1.42^b^	53.44 ± 1.50^a^
LDL	143.78 ± 4.36^a^	127.75 ± 4.62^a^	108.20 ± 4.14^b^	68.89 ± 4.36^c^
Triglycerides	150.78 ± 2.04^a^	140.88 ± 2.17^b^	126.20 ± 1.93^c^	115.00 ± 2.04^d^
Insulin	12.92 ± 0.36^a^	9.38 ± 0.38^b^	7.55 ± 0.35^c^	5.94 ± 0.37^d^

Note

The values are means ± *SD* of three independent determinations. PC (positive control without isoflavones); SIF_0.10_ (soy isoflavones: 0.10 g/kg body weight); SIF_0.15_ (soy isoflavones: 0.15 g/kg body weight); SIF_0.20_ (soy isoflavones: 0.20 g/kg body weight).

### 3.6 Insulin level

Effects of different levels of soy isoflavones on insulin level of PCOS induced rats are given in the Table 5. Significant reduction was observed in serum insulin level of all rats treated with SIF_0.10_, SIF_0.15,_ and SIF_0.20_, with the maximum reduction in SIF_0.20_ as 5.94 ± 0.37 (mg/dl) as compared to PC.

## 4 DISCUSSIONS

The purpose of this study was to investigate the effects of different levels of soy isoflavones on reproductive hormones, lipid profile, serum insulin, digestibility, and weight changes in polycystic ovarian syndrome (PCOS) induced female rats.

In this study, significant changes were observed in the levels of reproductive hormones after administration of soy isoflavones on different levels say SIF_0.10_, SIF_0.15,_ and SIF_0.20_ for 3 months. Significant increase in progesterone hormone was observed in all levels of soy isoflavones supplementation with maximum increase in SIF_0.20_ that is 13.21 ± 0.45 showing 30% increase from PC, whereas SIF_0.15_ and SIF_0.10_ showing 13% and 2% change only. Li et al., (2010) found similar result with 120 mg/day dosage of soy isoflavones after 8 weeks of supplementation. In PCOS, testosterone level increases because of the high levels of LH or high levels of insulin (Allahbadia & Merchant, 2011). This excessive testosterone causes other problematic issues like acne, hirsutism, and hair loss and also inhibits normal ovulation. So, reducing testosterone to the normal healthy level is the prime goal of PCOS treatment. And our study found statistically significant decrease in testosterone values in all treatment levels as 97.34 ± 3.03 (ng/dl) in SIF_0.10_, 89.29 ± 2.71 (ng/dl) in SIF_0.15,_ and 79.61 ± 2.85 (ng/dl) in SIF_0.20_. (Rajan & Balaji, 2017 and Khani et al., 2011) found similar results on decrease in testosterone levels by using different dosage levels of soy isoflavones for different time periods.

Moreover, in FSH/LH ratio, no statistically significant increase in FSH values was noted in SIF_0.10_ and SIF_0.15_, but a significant increase of 6.8% was observed in SIF_0.20_. Similar results were found by Forouhari et al., (2013) where no statistically significant change in FSH level was observed after 2 months of supplementation. But increase in FSH concentration in SIF_0.20_ was contradictory with all studies, might be this increase was a result of high dosage of soy isoflavone, whereas remarkable decrease was observed in LH values with lowest most observed in SIF_0.20_ as (13.91 ± 0.67 mIU/ml). Khani et al., (2011) suggested similar benefits by using 36 mg/day of soy isoflavones supplementation for 3 months in women having PCOS. LH lowering effects of soy isoflavones were also suggested in other studies (Cassidy et al., 1994; Hooper et al., 2009; Li et al., 2010; Yuan et al., 2012). Increase was observed in prolactin values from PC in both SIF_0.10_ and SIF_0.20_ levels; however, reduction was noted in SIF_0.15_ (31.93 ± 1.04 ng/ml) from PC. Similar findings were suggested by Li et al., (2010) after using 120 mg of soy isoflavones per day for 8 weeks. In estrogen concentration, significant increase of 46% was observed in SIF_0.20,_ but no statistically significant change was noted in SIF_0.10_ and SIF_0.15_ as compared to PC. Increase in estrogen levels was noted in a meta‐analysis of 47 studies on both pre‐ and postmenopausal women by Hooper et al., (2009), whereas many studies suggested significant decrease in estrogen level after different level of soy isoflavones administration (Kurzer, 2002 and Foth & Nawroth, 2003).

Dyslipidemia is a common problem in women with PCOS (Kim & Choi, 2013;). Combating with abnormal lipid profile is an important consideration in PCOS treatment. Our study showed **s**ignificant reduction in cholesterol, 14% in SIF_0.15_ and 22% in SIF_0.20_ as 141.60 ± 2.56 (mg/dl) and 127.56 ± 2.69 (mg/dl) while statistically insignificant results were obtained in SIF_0.10_ with 5% change as compared to PC. (Zhan & Ho, 2005; Taku et al., 2007) found similar results in total cholesterol reduction with soy isoflavones supplementation. Serum HDL concentration was significantly improved in all levels (SIF_0.10_, SIF_0.15_ and SIF_0.20)_ as 26.88 ± 1.59 (mg/dl), 32.40 ± 1.42 (mg/dl) and 53.44 ± 1.50 (mg/dl) in comparison with PC. Similarly significant decrease in LDL after 3 months of 36 mg/day genistein supplementation was observed by Khani et al., (2011). Significant reduction in serum LDL was noted as 68.89 ± 4.36 (mg/dl) in SIF_0.20_, and to 108.20 ± 4.14 (mg/dl) in SIF_0.15,_ whereas insignificant reduction was observed in SIF_0.10_ (127.75 ± 4.62 mg/dl) as compared to PC. The results of meta‐analysis by Zhan and Ho (2005) and Taku et al., (2007) showed similar reduction in LDL concentration after soy isoflavones supplementation. Overall, significant decrease was noted in triglycerides concentration, with highly significant in SIF_0.20_ as 115.00 ± 2.04 (mg/dl). However, significant reduction was observed in both SIF_0.10_ and SIF_0.15_ as compared to PC after 3 months soy isoflavone's supplementation. A significant reduction in triglycerides concentration after 50 mg/day of soy isoflavones intake for 12 weeks in 70 women with PCOS was suggested by Jamilian and Asemi (2016). Other studies by Jassi et al., (2010); Romualdi et al., (2008);; Zhan and Ho (2005) also found triglyceride improving effects of soy isoflavones supplementation.

Overall, significant reduction was noted in serum insulin level of all rats treated with SIF_0.10_, SIF_0.15,_ and SIF_0.20_, with the maximum reduction in SIF_0.20_ as 5.94 ± 0.37 (mg/dl) as compared to PC. Similar trial of 70 women with PCOS given 50 mg/day soy isoflavones for 12 weeks was conducted by Jamilian and Asemi (2016) found significant decreased in circulating serum levels of insulin homeostasis model of assessment estimated insulin resistance and increased quantitative insulin sensitivity check index. But soy isoflavones were found to have more potent effects on fasting insulin level (Aubertin‐Leheudre et al., 2008; Villa et al., 2009).

## 5 CONCLUSION

Our study revealed that soy isoflavones have potential role on reproductive hormones, insulin levels, weight, lipid profile, and nutrient digestibility in PCOS induced rats. Significant effects were observed on testosterone, LH, prolactin, estrogen, cholesterol, HDL, LDL, triglyceride, and insulin, whereas progesterone and FSH showed statistically significant results only in level SIF_0.20_; however, no effects were observed in lower dosage levels, might be due short duration of the study. Although significant results were found in high dosage level of soy isoflavones, nut long‐term administration of this level may cause toxicity. So, long‐term study with high dosage level of soy isoflavones is required for further investigation.

## CONFLICT OF INTEREST

The authors have no conflict of interest.

## Data Availability

The data that support the findings of this study are available from the corresponding author upon reasonable request.
